This article has been retracted.

# miR-599 Inhibits Vascular Smooth Muscle Cells Proliferation and Migration by Targeting TGFB2

**DOI:** 10.1371/journal.pone.0141512

**Published:** 2015-11-09

**Authors:** Baodong Xie, Chunfeng Zhang, Kai Kang, Shulin Jiang

**Affiliations:** Department of Cardiovascular Surgery, the Second Affiliated Hospital of Harbin Medical University, Harbin, Heilongjiang, China; Peking Union Medical College Hospital, CHINA

## Abstract

Aberrant proliferation and migration of vascular smooth muscle cells (VSMCs) play a crucial role in the pathogenesis of cardiovascular diseases including coronary heart disease, restenosis and atherosclerosis. MicroRNAs are a class of small, non-coding and endogenous RNAs that play critical roles in VSMCs function. In this study, we showed that PDGF-bb, as a stimulant, promoted VSMCs proliferation and suppressed the expression of miR-599. Moreover, overexpression of miR-599 inhibited VSMCs proliferation and also suppressed the PCNA and ki-67 expression. In addition, we demonstrated that ectopic expression of miR-599 repressed the VSMCs migration. We also showed that miR-599 inhibited type I collagen, type V collagen and proteoglycan expression. Furthermore, we identified TGFb2 as a direct target gene of miR-599 in VSMCs. Overexpression of TGFb2 reversed miR-599-induced inhibition of VSMCs proliferation and type I collagen, type V collagen and proteoglycan expression. In conclusion, our findings suggest miR-599 plays a crucial role in controlling VSMCs proliferation and matrix gene expression by regulating TGFb2 expression.

## Introduction

Cardiovascular diseases are a major cause of death worldwide and they include atherosclerosis, coronary artery disease (CAD), stroke, congestive heart failure, hypertension, myocardial infarction (MI)[1–4]. It is accepted that abnormal proliferation of vascular smooth muscle cells (VSMCs) is a critical event in the development of cardiovascular diseases [5–7]. However, their detail molecular mechanisms have not been fully illuminated.

MicroRNAs (miRNAs) are a class of small (18–24 nucleotides) non-coding and endogenous RNAs that modulate gene expression through binding to 3’UTR (3’ untranslated regions) of target mRNAs to lead to protein translational repression [8–12]. A lot of studies have demonstrated that miRNAs are involved in various cellular processes including cell development, growth, survival, differentiation, proliferation and apoptosis [13–16]. Increasing evidences also find that deregulated expression of miRNA is implicated in many cancers such as gastric cancer, osteosarcoma, hepatocellular carcinoma, lung cancer and colorectal cancer [17–22]. Recently, many evidences have also proved that miRNAs play critical role in the VSMCs function [23]. For example, Torella et al. demonstrated that miR-133 played important roles in VSMCs phenotypic switch in vivo and in vitro [24]. Wang et al. showed that miR-31 expression was increased in quiescent differentiated VSMCs and decreased in proliferative cells treated by serum starvation and platelet-derived growth factor [25]. Li et al. reported that miR-638 was a key molecule in regulating human VSMC proliferation and migration by targeting the NOR1/cyclin D pathway [26]. However, functions of miRNAs in VSMC are still less explored.

Otaegui et al. showed that miR-599 in peripheral blood mononuclear cell may be relevant at the time of relapse in multiple sclerosis patients [27]. Wojcicka et al [28]. showed that four microRNAs (miR-425,miR-155, miR-599 and miR-592) potentially targeted THRB transcript. However, the role of miR-599 in VSMCs was still unknown. In this study, we showed that PDGF-bb, as a stimulant, promoted VSMCs proliferation and suppressed the expression of miR-599. Moreover, overexpression of miR-599 inhibited VSMCs proliferation and also suppressed the PCNA and ki-67 expression. In addition, we demonstrated that ectopic expression of miR-599 repressed the VSMCs migration. We also showed that miR-599 inhibited type I collagen, type V collagen and proteoglycan expression. Furthermore, we identified TGFb2 as a direct target gene of miR-599 in VSMCs. Overexpression of TGFb2 reversed miR-599 induced inhibition of VSMCs proliferation and type I collagen, type V collagen and proteoglycan expression.

## Materials and Methods

### Ethics Statement

The protocol for our study was approved by the Ethical Committee of the Second Affiliated Hospital of Harbin Medical University.

### Cells Culture and Oligonucleotide Transfection

The VSMCs cell line was purchased from Cascade Biologics (Portland, OR) and kept in DMEM/F12 medium(Dulbecco’s modified Eagle’s medium; Invitrogen, Carlsbad, CA). miR-599 and scramble oligonucleotide was purchased from GenePharma (Shanghai, China) and transfected into the VSMCs used Lipofectamine 2000 (Invitrogen, Carlsbad, CA) according to the manufacturer’s information.

### qRT-PCR

Total RNA of the cell was extracted by using TRIzol reagent (Invitrogen, CA) following to the manufacturer’s information. The expression of miR-599 and TGFB2 was detected using qRT-PCR according to standard protocol on the Bio-Rad PCR system (Bio-Rad, CA). U6 snRNA was used as the control for miR-599 expression and GAPDH was used as the control. The primer sequence was shown as follows: miR-599 sense, 5’-GUUGUGUCAGUUUAUCAAAC-3’; antisense, 5’- CTCCATATCGCACTTTAATCTCTAACT-3’; GAPDH sense, 5'-GCACCGTCAAGGCTGAGAAC-3'; and GAPDH antisense, 5'-TGGTGAAGACGCCAGTGGA-3'.

### Luciferase Reporter Assay

Cells at about 75% confluences were transfected with the TGFB2 3’UTR luciferase reporter vector and MUT TGFB2 3’UTR vector. Luciferase activities were detected using a Dual-Luciferase Assay System (Promega, China) at 48 h post transfection. Luciferase data was normalized as Renilla luciferase activity.

### Cell Proliferation and Migration

Cells were tranfected with miR-599 mimics or scramble or co-transfected with miR-599 mimics and TGFB2 vector, respectively. Cell Counting kit 8 (CCK8, Dojindo, USA) was used to detect the cell proliferation following to the manufacture’s information. Wound-healing assay was performed to measure cell migration. A sterile plastic tip was used to scratch the cell layer when cell was reached 90% confluency. Photographic images were taken under a microscope at different time points.

### Western Blotting

Protein extraction was used RIPA lysis buffer (Beyotime Biotech, China). Protein lysates were separated by 10%SDS-PAGE (sodium dodecyl sulfate-polyacrylamide gel electrophoresis) and then transferred to polyvinylidene difluoride membrane (PVDF, Millipore, USA). Membrane was blocked with 5% bovine serum albumin, followed by incubation with primary antibody: type I collagen, type V collagen (dilutions 1: 2000,Sigma, USA) and proteoglycan (dilutions 1: 1000, Abcam, USA) and TGFb2 (dilutions 1: 2000, Abcam, USA). Membranes then incubated with HRP conjugated secondary antibody and the signal was measured using the ECL plus Kit (Pierce, USA).

### Statistics Analysis

Results were displayed as mean ± SD. The significance between two groups was used Student’s t test. The significance between more than two groups was used One-way ANOVA. P < 0.05 was indicated as significant.

## Result

### miR-599 Is Inhibited by PDGF-bb in VSMCs

As shown in the Fig 1A, PDGF-bb induced VSMCs proliferation in a time-dependent and dose-dependent manner (Fig 1B). Moreover, miR-599 was downregulated after PDGF-bb treatment (Fig 1C and 1D).

**Fig 1:** miR-599 is inhibited by PDGF-bb in VSMCs. (A) PDGF-bb can induce VSMCs proliferation at time-dependently. (B) PDGF-bb can induce VSMCs proliferation at dose-dependently. (C) The expression of miR-599 was measured by qRT-PCR. (D) The expression of miR-599 was measured by qRT-PCR. *p<0.05, **p<0.01 and ***p<0.001.

### miR-599 Suppressed VSMCs Proliferation and Migration

As shown in the Fig 2A, the expression of miR-599 was increased in VSMCs after tranfection of miR-599 mimic. Ectopic expression of miR-599 suppressed the VSMCs proliferation (Fig 2B). We also found that overexpression of miR-599 inhibited the mRNA and protein expression of PCNA in VSMCs (Fig 2C and 2D). Moreover, ectopic expression of miR-599 suppressed the mRNA and protein expression of ki-67 in VSMCs (Fig 2E and 2F) (S1 Fig). In addition, we showed that ectopic expression of miR-599 inhibited VSMCs migration (Fig 3).

**Fig 2:** miR-599 suppressed VSMCs proliferation. (A) The expression of miR-599 was measured by qRT-PCR. (B) CCK-8 analysis showed that overexpression of miR-599 suppressed VSMCs proliferation. (C) The mRNA expression of PCNA in VSMCs was measure by qRT-PCR. (D) The protein expression of PCNA in VSMCs was measure by western blot. (E) The mRNA expression of ki-67 in VSMCs was measure by qRT-PCR. (F) The protein expression of ki-67 in VSMCs was measure by western blot.*p<0.05 and ***p<0.001.

**Fig 3:** miR-599 suppressed VSMCs migration. Overexpression of miR-599 suppressed VSMCs migration. ***p<0.001.

### miR-599 Inhibited Matrix Gene Expression in VSMCs

Overexpression of miR-599 suppressed the type I collagen mRNA and protein expression (Fig 4A and 4B). In addition, miR-599 overexpression inhibited the mRNA and protein expression of type V collagen (Fig 4C and 4D). Moreover, ectopic expression of miR-599 inhibited proteoglycan mRNA and protein expression (Fig 4E and 4F) (S2 Fig).

**Fig 4:** miR-599 inhibited matrix gene expression in VSMCs. (A) Overexpression of miR-599 suppressed the type I collagen mRNA expression. (B) The protein expression of type I collagen in VSMCs was measure by western blot. (C) Overexpression of miR-599 suppressed the type V collagen mRNA expression. (D) The protein expression of type V collagen in VSMCs was measure by western blot. (E) Overexpression of miR-599 suppressed the proteoglycan mRNA expression. (D) The protein expression of proteoglycan in VSMCs was measure by western blot.

### TGFb2 Is a Direct Target of miR-599 in VSMCs

TargetScan algorithms found that there was a potential seed sequence of miR-599 in the 3’UTR of TGFb2 (Fig 5A). We demonstrated that miR-599 inhibited the luciferase activity in the TGFb2 with wild-type 3’UTR, whereas, luciferase activity was not drop in the mutant binding sites 3’UTR of TGFb2 (Fig 5B). Overexpression of miR-599 suppressed the protein expression of TGFb2 (Fig 5C) (S3 Fig).

**Fig 5:** TGFb2 is a direct target of miR-599 in VSMCs. (A) There is a potential seed sequence of miR-599 in the 3’UTR of TGFb2. (B) miR-599 inhibited the luciferase activity in the TGFb2 with wild-type 3’UTR, whereas, luciferase activity was not drop in the mutant binding sites 3’UTR of TGFb2. (C) Overexpression of miR-599 suppressed the protein expression of TGFb2. ***p<0.001.

### TGFb2 Involved in the Effect of miR-599 in VSMCs

Western blot showed that the plasmid of TGFb2 promoted the TGFb2 protein expression (Fig 6A). CCK8 analysis demonstrated that overexpression of TGFb2 promoted miR-599-induced inhibition of VSMCs proliferation (Fig 6B). Moreover, ectopic expression of TGFb2 promoted the expression of type I collagen, type V collagen and proteoglycan in miR-599 overexpressing VSMCs (Fig 6B, 6C and 6D) (S4 Fig).

**Fig 6:** TGFb2 involved in the effect of miR-599 in VSMCs. (A) The protein expression of TGFb2 was measured by western blot. (B) Overexpression of TGFb2 promoted miR-599-induced inhibition of VSMCs proliferation. (C) Ectopic expression of TGFb2 promoted the expression of type I collagen, in miR-599 overexpressing VSMCs. (D) The mRNA expression of type V collagen in VSMCs was measure by qRT-PCR. (E) The mRNA expression of proteoglycan in VSMCs was measure by qRT-PCR. *p<0.05, **p<0.01 and ***p<0.001.

## Discussion

In this study, we showed that PDGF-bb, as a stimulant, promoted VSMCs proliferation and suppressed the expression of miR-599. Moreover, overexpression of miR-599 inhibited VSMCs proliferation and also suppressed the PCNA and ki-67 expression. In addition, we demonstrated that ectopic expression of miR-599 repressed the VSMCs migration. We also showed that miR-599 inhibited type I collagen, type V collagen and proteoglycan expression. Furthermore, we identified TGFb2 as a direct target gene of miR-599 in VSMCs and overexpression of TGFb2 reversed miR-599 induced inhibition of VSMCs proliferation and type I collagen, type V collagen and proteoglycan expression. Above findings suggest miR-599 plays a crucial role in controlling VSMCs proliferation and matrix gene expression.

Aberrant VSMCs proliferation and migration were associated with the development of cardiovascular diseases such as restenosis and atherosclerosis [26, 29, 30]. Accumulating studies indicated that miRNAs play an important role in a lot of cellular processes including cell differentiation, proliferation, epithelial—mesenchymal transition, migration and invasion [31–34]. Otaegui et al. showed that miR-599 in peripheral blood mononuclear cell may be relevant at the time of relapse in multiple sclerosis patients [27]. Wojcicka et al [28]. showed that four microRNAs (miR-425,miR-155, miR-599 and miR -592) potentially targeted THRB transcript. However, the role of miR-599 in VSMCs was still unknown. In our study, we confirmed that miR-599 was decreased in proliferative VSMCs induced by PDGF-bb. Overexpression of miR-599 suppressed VSMCs proliferation and migration and also inhibited the PCNA and ki-67 expression. We also showed that miR-599 inhibited type I collagen, type V collagen and proteoglycan expression.

TGF-b pathway plays an important role in many cellular processes such as cell differentiation, proliferation, extracellular matrix accumulation, tissue repair, inflammatory responses and immune [35–39]. TGF-b has three isoforms including TGF-b1, TGF-b2 and TGF-b3 in mammals [40]. Previous studies proved that TGF-b acted as important roles in the development in cardiovascular diseases such as atherosclerosis and restenosis [40, 41]. TGF-b stimulates cell proliferation and invasion, synthesis of extracellular matrix proteins and proteoglycans in VSMCs [41, 42]. In this study, we demonstrated that miR-599 acted as an important regulator by targeting TGF-b2 in VSMCs. TargetScan algorithms demonstrated there was a potential seed sequence of miR-599 in the 3’UTR of TGFb2. We further confirmed that miR-599 directly bound the 3’-UTR regions of TGFb2. Moreover, overexpression of miR-599 suppressed the expression of TGFb2 in VSMCs. Furthermore, overexpression of TGFb2 reversed miR-599 induced inhibition of VSMCs proliferation and type I collagen, type V collagen and proteoglycan expression.

In conclusion, we initially demonstrated that the expression of miR-599 was decreased in proliferating VSMCs treated by PDGF-bb. Overexpression of miR-599 suppressed VSMCs proliferation and migration and inhibited the PCNA and ki-67 expression. We also showed that miR-599 inhibited type I collagen, type V collagen and proteoglycan expression. Furthermore, we identified TGFb2 as a direct target gene of miR-599 in VSMCs and overexpression of TGFb2 reversed miR-599 induced inhibition of VSMCs proliferation and type I collagen, type V collagen and proteoglycan. These findings suggest miR-599 plays a crucial role in controlling VSMCs proliferation and matrix gene expression by regulating TGFb2 expression.

## Supporting Information

S1 Fig The protein expression of PCNA and ki-67 was shown. (TIF)

S2 Fig The protein expression of type I collagen, type V collagen and proteoglycan was shown. (TIF)

S3 Fig The protein expression of TGFb2 was shown. (TIF)

S4 Fig The protein expression of TGFb2 was measured by Western blot analysis after treated with plasmid of TGFb2. (TIF)
